The article "Risk factors for postoperative complication after spinal fusion and instrumentation in degenerative lumbar scoliosis patients" was published in 2014. Journal: J Orthop Surg Res.

# Risk factors for postoperative complication after spinal fusion and instrumentation in degenerative lumbar scoliosis patients

**DOI:** 10.1186/1749-799X-9-15

**Published:** 2014-03-07

**Authors:** Honghui Tang, Jianfei Zhu, Feng Ji, Shouguo Wang, Yue Xie, Haodong Fei

**Affiliations:** 1 Department of Orthopedics, Huai'an First People's Hospital, Nanjing Medical University, 6 Beijing Road West, Huai’an, Jiangsu 223300, People's Republic of China; 2 Department of Orthopedics, The 82nd Hospital of PLA, Huai’an 223300, People's Republic of China

**Keywords:** Degenerative lumbar scoliosis, Postoperative complications, Predictive factors, Spinal fusion

## Abstract

**Background:**

Relatively few studies have focused on the major medical complications that are more common in older adults. Furthermore, these studies have generally not reported how accurately a risk factor, or combination of risk factors, can distinguish between those who will have a complication and those who will not.

**Methods:**

A total of 236 consecutive patients who had undergone surgical treatment for degenerative lumbar scoliosis between June 2008 and June 2012 were included retrospectively in this study. The demographic distribution, medical history, and clinical data were collected to investigate the predictive factors of postoperative complications by logistic regression.

**Results:**

Among 236 eligible patients, major medical complications occurred in 7.2% of cases and wound complications occurred in 1.7% of cases. Ninety-day mortality rate was 0.4%. Postoperative complications were strongly associated with history of severe chronic obstructive pulmonary disease (COPD) (*P* = 0.031), dyspnea with minimal exertion (*P* = 0.041), being at least partially dependent (*P* = 0.041), smoking within the past year (*P* = 0.044), American Society of Anesthesiologists (ASA) class of more than 2 (*P* = 0.000), diabetes treated with insulin (*P* = 0.003), and steroid use for chronic condition (*P* = 0.003). In logistic regressions, operation time (odds ratio 2.45, 95% confidence interval 1.11–4.78), ASA class (class 3 or 4 vs. class 1 or 2: odds ratio 2.21, 95% confidence interval 1.22–3.45), insulin-dependent diabetes (odds ratio 1.72, 95% confidence interval 1.18–2.43), and steroid use for chronic condition (odds ratio 1.55, 95% confidence interval 1.06–2.32) may be reasonable predictors for an individual's likelihood of surgical complications.

**Conclusions:**

The occurrence of postoperative complications is most likely multifactorial and is related to operation time, ASA class, insulin-dependent diabetes and steroid use for chronic condition.

## Introduction

The identification and quantification of risk factors for postoperative complication after spine surgery are of paramount importance to the patient and the clinician. This concern is especially important among older patients, in whom complications are more common than among younger adults. In addition to its obvious importance for patient safety, risk factor information becomes critical as health care policy makers implement and enforce ‘quality’ metrics.

The article "Risk factors for postoperative complication after spinal fusion and instrumentation in degenerative lumbar scoliosis patients" was published in 2014. Journal: J Orthop Surg Res.

Degenerative lumbar scoliosis is a common diagnosis prompting spine surgery in older adults, and surgical rates have increased in this population [1]. Other studies of spine surgery complications have often focused on general populations, all diagnoses, or other single conditions rather than on older adults with degenerative scoliosis [2-4]. Many studies have only focused on complications during the surgical hospitalization or on specific types of complications, such as device complications or infections [5,6]. Relatively few studies have focused on the major medical complications that are more common in older adults. Furthermore, these studies have generally not reported how accurately a risk factor or combination of risk factors can distinguish between those who will have a complication and those who will not.

This retrospective cohort study was undertaken to investigate (1) the incidence of postoperative complication in a larger degenerative lumbar scoliosis population treated with spinal fusion and instrumentation and (2) the predictive factors of development of postoperative complication after spine surgery in unselected degenerative lumbar scoliotic patients who underwent spinal surgery.

## Materials and methods

A total of 236 consecutive patients (from the Spine Unit of the authors' hospital) who had undergone surgical treatment for degenerative lumbar scoliosis between June 2008 and June 2012 were included retrospectively in this study. Inclusion criteria were minimum age at surgery of 40 years, Cobb angle of more than 10° before surgery, and minimum 1-year follow-up. Exclusion criteria included diagnosis of scoliosis with other etiologies (idiopathic, paralytic/neuromuscular, or congenital) and age of less than 40 years at the time of surgery. They included 81 men and 155 women ranging in age from 47 to 77 years with a mean of 61.7 years. When the patients sought medical treatment in our hospital for the first time, the duration of disease ranged from 4 months to 17 years with a mean of 5.2 years. Main clinical manifestations were low back pain, radiculopathy, and claudication. Preoperative assessment included routine lumbar posterior-anterior and flexion-extension position radiographs, lumbar computed tomography (CT) and magnetic resonance imaging (MRI) in all patients, and lumbar myelography in some patients to ascertain whether there was complicated lumbar intervertebral disc protrusion, canal stenosis, or spondylolisthesis. Most patients (95%) underwent conservative treatment which included bed rest, administration of non-steroidal anti-inflammatory drugs, avoidance of lifting heavy objects, and other changes in lifestyle for about 6 months before surgery. When all these treatments failed to work effectively and symptoms deteriorated, surgical intervention was performed. In patients (5%) who had severe symptoms of canal stenosis or nerve root compression, especially cauda equina syndrome, when they first visited the clinic, surgical treatment was the initial form of management. A total of 21 patients with postoperative complications were identified, and scoliotic patients without postoperative complications were chosen and best matched for sex, age, approximate date of surgery, and diagnosis with patients with postoperative complications at a 4:1 ratio, respectively.

The article "Risk factors for postoperative complication after spinal fusion and instrumentation in degenerative lumbar scoliosis patients" was published in 2014. Journal: J Orthop Surg Res.

Surgical modalities were dependent on the clinical symptoms and imaging findings. In our series, simple nerve root decompression was performed in 13 cases whose main clinical presentation was nerve root symptoms without lower back pain, intermittent claudication, or significant canal stenosis; decompression by posterior laminectomy plus bone graft fusion of short (≤3 segments) or long (>3 segments) fixation with pedicle screw instrumentation was performed in the other 92 patients. The latter surgical modality was used mainly for degenerative lumbar scoliosis complicated by intervertebral disc protrusion, canal stenosis, and instability or spondylolisthesis of the lumbar vertebrae. Short fusion and fixation was mainly used in patients with local/sectional intraspinal nerve compression and without obvious symptoms of instability and nerve compression in the upper and lower vertebral segments, especially for those in poor condition who could not tolerate significant trauma. Long fusion and fixation was mainly used in patients with multisegmental neural compression and/or spinal instability. Intervertebral fusion, posterolateral fusion, or interlaminar fusion was performed after fixation.

In those patients who had American Society of Anesthesiologists (ASA) class of more than 2, special anesthetic regimens such as central venous line access and arterial blood pressure monitoring were utilized. In all patients, a Cell Saver system (Haemonetics, Braintree, MA, USA) was used intraoperatively to reinfuse shed blood. The volume of blood collected by the Cell Saver system was recorded, and estimated blood loss was calculated by measuring loss through Cell Saver suction and by weighing the surgical sponges. The surgery was performed on the patient under hypotensive anesthesia in which systolic blood pressure was kept to <90 mmHg. The same blood transfusion and prophylactic antibiotic guidelines were used for all patients. Allogenic blood transfusion was performed if hemoglobin decreased to <7.0 mg/dL or if anemic symptoms developed, such as a decrease in blood pressure to <100 mmHg systolic, tachycardia >100 beats/min, or a low urine output of <30 mL/h, even after initial fluid challenge with 500 mL of normal saline in patients with a hemoglobin level between 7.0 and 8.0 mg/dL [7,8]. All patients were given a dose of 1 g first-generation cephalosporin 30 min before skin incision and were covered for 24 h with three additional doses. For the patients with steroid use for chronic condition in the perioperative period (patient on 10–25 mg of prednisolone per day, patient stopped oral steroids of >10 mg prednisolone per day within last 3 months, or patient on inhaled steroids of >1.5 mg beclomethasone or 750 μg flixotide per day), we use the regiment of 25 mg hydrocortisone IV on induction, 25 mg hydrocortisone IV QDS for 48–72 h, and then normal steroids postoperation.

The article "Risk factors for postoperative complication after spinal fusion and instrumentation in degenerative lumbar scoliosis patients" was published in 2014. Journal: J Orthop Surg Res.

Information was compiled about perioperative complications occurring within 30 days after the operation. This information included both surgical (postoperative bleeding, wound breakdown, return to operating room, infection, implant failure, neurological compromise, and others) and non-surgical complications (pulmonary disease, arrhythmia, hemodynamic instability requiring inotropic support, deep vein thrombosis (DVT), pulmonary embolism, and others). All patients had a minimum of 1 year of follow-up. Follow-up data collected included postoperative Cobb angle, unanticipated late reoperation, and other complications.

The approval of the institutional ethics committee was obtained (no. 20120121). Factors associated with the occurrence of postoperative complications were identified using univariate analysis. The data analysis was performed using SPSS (version 19.0, IBM, Armonk, NY, USA). Continuous data were compared between the patients with postoperative complications and control groups using Student's *t* test, whereas discontinuous data were analyzed using the chi-square test. The Fisher exact test was used for small data subsets (*n* < 5). All significance tests were two-tailed, with *P* < 0.05 representing statistical significance.

## Results

### Demographic data

A summary of the clinical data before spinal fusion for the patients with postoperative complications and control groups (those without postoperative complications) is presented in Table 1. Of the 21 patients identified as having postoperative complications, 10 had history of severe chronic obstructive pulmonary disease (COPD) (47.6%), 5 had dyspnea with minimal exertion (23.8%), 7 were at least partially dependent (33.3%), 12 were smoking within the past year (57.1%), 18 had ASA class of more than 2 (75.7%), 15 had diabetes treated with insulin (71.4%), and 12 had steroid use for chronic condition (57.1%). An additional 84 patients without postoperative complications matched for age, diagnosis, and year of surgery also were evaluated. Of the patients in the control group, 20 had history of severe COPD (23.8%), 6 had dyspnea with minimal exertion (7.1%), 10 were at least partially dependent (11.9%), 28 were smoking within the past year (33.3%), 31 had ASA class of more than 2 (36.9%), 26 had diabetes treated with insulin (31.0%), and 20 had steroid use for chronic condition (23.8%). No significant differences were observed between the two groups in age, sex ratio, and body mass index (BMI). The strong risk factors for the development of postoperative complications were history of severe COPD (*P* = 0.031), dyspnea with minimal exertion (*P* = 0.041), being at least partially dependent (*P* = 0.041), smoking within the past year (*P* = 0.044), ASA class of more than 2 (*P* = 0.000), diabetes treated with insulin (*P* = 0.003), and steroid use for chronic condition (*P* = 0.003).

The article "Risk factors for postoperative complication after spinal fusion and instrumentation in degenerative lumbar scoliosis patients" was published in 2014. Journal: J Orthop Surg Res.

**Table 1:** Demographic characteristics, functional status, and health habits of the patientss

**Characteristics**	**Patients with postoperative complications**		***P***
	**Yes (*n*** **= 21)**	**No (*n*** **= 84)**	
Age (years)	66.8 ± 5.5	65.0 ± 5.1	0.166
Sex			0.324
Male	5 (23.8)	12 (14.2)	
Female	16 (76.2)	72 (85.8)	
BMI (kg/m^2^)	26.8 ± 2.3	25.8 ± 3.2	0.183
History of severe COPD			0.031
Yes	10 (47.6)	20 (23.8)	
No	11 (52.4)	64 (76.2)	
Dyspnea with minimal exertion			0.041
Yes	5 (23.8)	6 (7.1)	
No	16 (76.2)	78 (92.9)	
Functional health status			0.041
Independent	14 (66.7)	74 (88.1)	
At least partially dependent	7 (33.3)	10 (11.9)	
Smoker within past year			0.044
Yes	12 (57.1)	28 (33.3)	
No	9 (42.9)	56 (66.7)	
ASA class			0.000
1 or 2	3 (14.3)	53 (63.1)	
3	16 (76.2)	27 (32.1)	
4	2 (9.5)	4 (4.8)	
Diabetes			0.003
None or diet only	3 (14.3)	28 (33.3)	
Oral agents	3 (14.3)	30 (35.7)	
Insulin	15 (71.4)	26 (31.0)	
Steroid use for chronic condition			0.003
Yes	12 (57.1)	20 (23.8)	
No	9 (42.9)	64 (76.2)	

Note: BMI: body mass index; COPD: chronic obstructive pulmonary disease; ASA indicates American Society of Anesthesiologists.

### Operative data

The average forced vital capacity (FVC) before operation was less in patients with postoperative complications than in those without postoperative complications, 69.8% ± 10.4% versus 73.9% ± 7.5% (*P* = 0.042). Number of levels fused was 4.2 ± 0.8 versus 3.7 ± 1.0 (*P* = 0.029). Operation time was 296.5 ± 51.4 min versus 217.7 ± 46.8 min (*P* = 0.000). Estimated blood loss was 999.8 ± 218.1 mL versus 849.3 ± 275.6 mL (*P* = 0.022), respectively. Of the 21 patients with postoperative complications, 12 patients (57.1%) received allogenic blood perioperatively, either as red blood cells or whole blood. On average, 2.3 ± 2.0 units per patient (U/pt) was given perioperatively. However, in the control group, 29 patients (34.5%) received allogenic blood transfusion perioperatively, either as red blood cells or whole blood. On average, 1.5 ± 1.1 U/pt was given perioperatively. The use of allograft was not statistically associated with increased risk of infection: It was used in 15 of 21 in the group with infection, as compared with 50 of 84 in the uninfected matched cohort (*χ*^2^*P* = 0.315) (Table 2).

The article "Risk factors for postoperative complication after spinal fusion and instrumentation in degenerative lumbar scoliosis patients" was published in 2014. Journal: J Orthop Surg Res.

**Table 2:** Predictive factors for the postoperative complications

**Characteristics**	**Patients with postoperative complications**		
	**Yes (*n*** **= 21)**	**No (*n*** **= 84)**	***P***
FVC (%)	69.8 ± 10.4	73.9 ± 7.5	0.042
Surgical Procedure, *n* (%)			0.458
Decompression alone	1 (4.8%)	12 (14.3%)	
Instrumented fusion	20 (95.2%)	72 (85.7%)	
No. of levels fused	4.2 ± 0.8	3.7 ± 1.0	0.029
Op time (min)	296.5 ± 51.4	217.7 ± 46.8	0.000
EBL(mL)	999.8 ± 218.1	849.3 ± 275.6	0.022
Transfusion( U/pt)	2.3 ± 2.0	1.5 ± 1.1	0.022
Allograft, *n* (%)			0.315
Yes	15 (71.4%)	50 (59.5%)	
No	6 (28.6%)	34 (40.5%)	

Note: FVC: forced vital capacity; Op time: operation time; EBL: estimated blood loss during operation; U blood units: U/pt: units per patient.

### Overall complication rates

Our combined variable for major medical complications occurred in 7.2% of cases, and wound complications occurred in 1.7% of cases. Ninety-day mortality rate was 0.4%. Among major medical complications, bleeding requiring >4 units of RBCs was the most common, followed by pneumonia and DVT/thrombophlebitis (Table 3).

**Table 3:** Overall complication rates for patients underwent surgery for lumbar degenerative scoliosis, 2008-2012 (N = 236)

**Complication**	**n**
Return to operating room	2
Urinary tract infection	2
Death within 90 d	1
Congestive heart failure in 1 mo after surgery	1
Progressive renal insufficiency	1
Acute renal failure	1
Peripheral nerve injury	3
Bleeding requiring > 4 units of RBCs	7
Pneumonia	5
Reintubation for respiratory or cardiac failure	2
Myocardial infarction	1
Failure to wean > 48 hr	1
DVT/thrombophlebitis	4
Pulmonary embolism	1
Cerebrovascular accident/stroke	1
wound complication	4

Total number of patients in these composites is not the sum of individual complications because some patients had more than 1 complication. RBC indicates red blood cell; CPR, cardiopulmonary resuscitation; DVT, deep vein thrombosis.

The article "Risk factors for postoperative complication after spinal fusion and instrumentation in degenerative lumbar scoliosis patients" was published in 2014. Journal: J Orthop Surg Res.

### Predictive factors of postoperative complications

In the postoperative complications group, by multivariate logistic regression analysis, operation time, ASA class, insulin-dependent diabetes, and steroid use for chronic condition were identified to be factors that remained statistically significant (*P* < 0.05) in predicting the probability of postoperative complications (*R*^2^ = 0.668) (Table 4).

**Table 4:** Multivariate regression model of predicting postoperative complications after surgery for degenerative lumbar scoliosis

**Predictors**	**Odds ratio**	**95% confidence Interval**		***P *** **values**
		**Lower limit**	**Upper limit**	
Operation time	2.45	1.11	4.78	0.001
ASA class (more than 2)	2.21	1.22	3.45	0.003
Insulin	1.72	1.18	2.43	0.023
Steroid use for chronic condition	1.55	1.06	2.32	0.031

Nagelkerke R^2^ = 0.668.

## Discussion

In this older, largely adult degenerative lumbar scoliosis patient population, more than 5% had major medical complications or 90-day mortality. This emphasizes the importance of studying major medical complications of degenerative lumbar scoliosis surgery, in addition to wound complications and device complications. Our results also indicate that in contrast to BMI, preoperative FVC, surgical procedure, operation time and other clinical characteristics, number of levels fused, ASA class, insulin-dependent diabetes, and steroid use for chronic condition were best predictors of major medical complications after surgery for degenerative lumbar scoliosis.

It is well established in spine surgery that insulin-dependent diabetes predisposes patients to postoperative complications [9]. Richard et al. [10] found insulin-requiring diabetes as a better predictor of complications compared with diabetes controlled with diet or oral agents alone. The results of the present study demonstrate that insulin-using diabetic patients were more likely to suffer from postoperative complications than non-insulin-using diabetic patients in the postoperative period (adjusted risk ratio = 1.72, 95% confidence interval 1.18–2.43). A possible explanation may be that patients with insulin-dependent diabetes might have more serious and wider array of systemic manifestations than non-insulin-dependent diabetes patients. On the basis of these data, it seems prudent to warn insulin-dependent diabetic patients of the potential increased risk of postoperative complications associated with degenerative lumbar scoliosis surgery. When insulin-dependent diabetic patients do require lumbar instrumentation and fusion procedures, adjunctive measures, such as thorough preoperative medical evaluation and aggressive perioperative medical management, should be undertaken.

The article "Risk factors for postoperative complication after spinal fusion and instrumentation in degenerative lumbar scoliosis patients" was published in 2014. Journal: J Orthop Surg Res.

Patients with high preoperative ASA levels have been documented to be associated with higher morbidity and mortality rates in spinal surgery [11,12]. Veeravagu et al. [11] analyzed 24,774 patients who underwent a spinal decompression and fusion between 1997 and 2006 from the Veterans Affairs' National Surgical Quality Improvement Program database and reported ASA class of 3 (OR = 1.45) or 4 to 5 (OR = 1.66) as a statistically significant predictor of postoperative infection. Pateder [12] came to a similar conclusion in another series of 361 adults with spinal deformity who underwent 407 corrective procedures, in which the average preoperative ASA levels for patients who died and patients who survived were 3.0 and 2.3, respectively (*P* < 0.0001). They concluded that there was a strong association between increasing ASA class and increasing mortality. In line with the studies of Veeravagu et al. and Pateder et al., our study demonstrated that a preoperative ASA class of ≥3 was the most accurate indicator for an increased risk for a major complication, suggesting that spinal fusion should be carefully considered in degenerative lumbar scoliosis patients whose preoperative ASA class is more than 2.

It has been previously suggested that prolonged operative time was associated with an increased prevalence of postoperative spinal wound complications [13,14]. The results of the present study demonstrate that patients with longer surgical time were more likely to suffer from delayed infections in the postoperative period (adjusted risk ratio = 2.45, 95% confidence interval 1.11–4.78). A possible explanation may be that contamination of the sterile field occurs during the extended preoperative setup time. Possible contamination sources include direct contact with the sterile field, airborne contamination from traffic [15], or loss of sterile technique. Dalstrom et al. [16] conducted a study in a simulated operating room environment and found a significant correlation between the length of time that the sterile tray is exposed to the air and the contamination rate of the instruments. Covering the tray with a sterile towel after it is opened reduces this contamination risk. The other strength of this study is that we included a large cohort of patients with degenerative lumbar scoliosis surgeries.

Kelly et al. [17] reported that chronic steroid use was one of the major predictors of 30-day readmissions in major gastrointestinal resections. Malviya et al. [18] also came to a conclusion that prolonged corticosteroid use has a negative influence upon the long-term implant survival. They hypothesized that the potential causes might include the deleterious influence on bone ingrowth and osteopenia resulting in a risk of fracture. In our study, we found that patients with chronic steroid use were 1.55 times as likely to have postoperative complications as those without. This association may reflect the effects of steroids on wound healing and recovery, but is likely a marker for underlying chronic disease, inflammation, and additional comorbidities.

The article "Risk factors for postoperative complication after spinal fusion and instrumentation in degenerative lumbar scoliosis patients" was published in 2014. Journal: J Orthop Surg Res.

The findings of this study should be viewed after considering the following limitations. Firstly, these data represent the experience at as single institution that is an academic tertiary care center with trainees in the anesthesia, orthopedic, neurosurgical, and nursing departments. Secondly, our data collection system only captured wound infection information on patients who returned to our hospital for treatment. Patients with localized superficial infections who were managed successfully as an outpatient would not be included in this study. However, we consider these infections to be clinically significant as these patients required further hospitalization and/or additional surgeries to treat their infections. Moreover, the results are limited by a relatively small sample size and the broad time period covered. In addition, changes in anesthetic and surgical practices over time may have affected patient outcomes. Finally, we also acknowledge the limitations introduced by our patients' clinical heterogeneity.

## Conclusion

In conclusion, the risks for postoperative complications after surgery for degenerative lumbar scoliosis are multifactorial. Multivariate logistic regression analysis suggest that operation time, ASA class, insulin-dependent diabetes, and steroid use for chronic condition may be reasonable predictors for an individual's likelihood of surgical complications. Such prediction rules might improve surgical planning, the patient consent process, and strategies for reducing risk.

## Competing interests

The authors declare that they have no competing interests.

## Authors’ contributions

The design of the study was done by JF. TH and ZJ prepared the manuscript and assisted in the study processes. WS, XY, and FH assisted in the data collections. All authors read and approved the final manuscript.
